The article "Application of Nanocellulose Biofilter from Pineapple Peel Waste for Water Microbes Removal" was published in 2023. Journal: J Environ Public Health.

# Application of Nanocellulose Biofilter from Pineapple Peel Waste for Water Microbes Removal

**DOI:** 10.1155/2023/5823207

**Published:** 2023-01-28

**Authors:** Rini, Heru Suryanto, Purnama Dini Hari, Daimon Syukri, Jaswandi, Fredy Kurniawan, Muhammad Makky

**Affiliations:** ^1^Department of Food and Agricultural Product Technology, Andalas University, Padang, Indonesia; ^2^Department of Mechanical Engineering, Malang State University, Malang, Indonesia; ^3^Department of Animal Production, Andalas University, Padang, Indonesia; ^4^Department of Chemistry, Faculty of Science and Data Analytics, Institut Teknologi Sepuluh Nopember, Surabaya, Indonesia; ^5^Department Agricultural Engineering and Biosystem, Andalas University, Padang, Indonesia

## Abstract

This research aimed to assess the effectiveness of nanocellulose biofilter (NCB) made from pineapple peel waste to reduce the number of microbes in water. Further processing of cellulose from nata de pina into nano size was proposed, then transformed into a filter membrane. Three types of NCB were developed: bacterial cellulose acetate membrane, bacterial cellulose acetate membrane with TiO_2_ treatment, and bacterial cellulose acetate membrane with TiO_2_ and graphite nanoplatelet treatment. These NCBs were used to filter microbes in several water sources in Padang City, West Sumatra Province. The filtering process was carried out using a filter holder where the NCB had been installed. The number of microbes contained in the water, including *E. Coli*, was determined before and after filtering. As a result, all NCBs reduced the total microbes in water by about 50%. Furthermore, when applied to water pollutant bacteria, *E. Coli*, all prepared NCBs reduced them by more than 90%. The effectiveness of all NCBs to remove microbes' contamination, especially bacteria, looks very promising with or without TiO_2_ and graphene reinforcement. Although the efficacy of all NBC for microbial water purification was relatively similar, further experiments to clarify the superior of TiO_2_ and graphite nanoplatelet on NCB need to be carried out, especially in reducing chemical contamination.

## 1. Introduction

Cellulose fiber as a polymer matrix has developed rapidly in the last decade [1]. Its advantages include good mechanical properties, low density, environmentally friendly, abundant abundance, inexpensive, nontoxic, easily degraded, and included in renewable natural resources. Cellulose fibers can be produced from plants, marine animals, and bacteria. Using forest plants to create cellulose fibers continuously has significantly reduced Indonesia's area and forest resources. This results in forest destruction, soil erosion, floods, landslides, and global warming. To minimize the negative impact caused by the cellulose production of these plants, it is necessary to find other alternatives to produce cellulose fiber. Using agricultural waste is one solution to obtain cellulose-producing materials [2].

Numerous experiments have been attempted to create nanocellulose from sources of fiber besides wood, such as agricultural waste [3]. Wheat straws, corn cobs, pineapple leaves, soybean shells, bagasse, pineapple peel, and other agricultural wastes can be used to manufacture nanocellulose. The pineapple peel waste is one of the agricultural wastes with a significant amount of potential for development as a source of nanocellulose raw materials. This is a result of Indonesia's extensive pineapple output. In Indonesia, there are more than 28,000 hectares of pineapple farms. With a 23% pineapple peel waste percentage and an annual production rate of 20 tons of pineapple per hectare, more than 128,000 tons of pineapple peel trash are produced. This has a great deal of development potential [4–6].

Pineapple peel waste can be developed into a nanocellulose biomembrane, which can be used as an auxiliary medium in water purification [7]. In general, water pollution by microbes is a pollution that has an excellent potential to occur. In contrast to chemical pollution that may arise if there is the use of chemicals around water bodies or poor soil conditions, microbiological pollution is very susceptible to occur because water is a substance that becomes a medium for microbial growth. Membranes are becoming prevalent in the wastewater treatment, especially domestic waste. This is due to the remarkable efficiency of the technology in reducing the pollution level in wastewater. Other benefits include minimal energy consumption, less need for additional chemicals during operation to prevent more waste production, ease of operation and maintenance, and less land requirement [8, 9].

In this study, the development of bacterial nanocellulose from pineapple peel as the raw material of a nanocellulose biofilter was proposed due to its green production, which could avoid the multipurification process involving harsh chemicals and time-consuming [10]. As a membrane biofilter, the NCB works to separate different substances by allowing some to pass while others are stopped due to the microstructure and chemistry of the membrane material. The NBC was designed with well-defined pores for size exclusion and tailored surface chemistry with TiO_2_ and graphite nanoplatelet to strengthen the selective adsorption of a specific contaminant. Several developed NCBs were applied for microbes' removal in water to enhance the primary data for developing biomembranes made from agricultural waste that can positively impact the community in the future. The water used in this research was collected in Padang, where industrial pollution is still low [11]. Only domestic pollutants, which may have considerable microbial contamination, are the subject of current research.

## 2. Material and Method

### 2.1. NCB Preparation

#### 2.1.1. Bacterial Cellulose Synthesis

The schematic of the experiment is described in Figure 1. According to Retegi et al. (2010), the experiment was started by producing bacterial cellulose with some modifications [12]. The bacterial cellulose synthesis began with the making of nata from the juice of pineapple peel. The bacteria used in the step were *Acetobacter xylinum*. A 5 kg pineapple peel was washed thoroughly and cut into small pieces. After that, the parts of the pineapple peel were ground and filtered to extract the juice. 10 L of the juice was cooked and then added with 10% (w/v) of granulated sugar, 0.5% (w/v) of ammonium sulfate, and diluted acetic acid to adjust the acidity to pH 4.5. Furthermore, the boiled mixture solution was cooled at room temperature. The culture media was then put into plastic containers. The bacterial starter material was added as much as 20%, covered with aluminium foil, tied with rubber, and fermented for ten days to produce nata de pina.

The high-pressure homogenizer (HPH) process was conducted to reduce the pore size of produced bacterial cellulose (BC). The cellulose sheets from the previous process were washed repeatedly using water until neutral (pH 7) and the outer layer is cleaned. Then, the BC pellicle was purified by immersing it in a solution of 1% NaOH. Twenty-four hours later, it was washed with water until the pH was neutral. After that, the BC was cut into small pieces and then pulverized using a blender machine with a speed of 2600 rpm for 5 minutes and mixed 250 ml of cellulose with 750 ml of distilled water. The mixture was then homogenized using HPH with five repetition cycles at a pressure of 150 bar. The solution was then filtered, and the nanocellulose solution was poured into plastic-coated glass moulds and dried in an oven at 60°C for 8 h.

#### 2.1.2. Nanocellulose Biofilter (NCB) Production

The preparation of NCB from the pineapple peel was conducted according to the previous research. The preparation of cellulose acetate refers to the Coba method [13]. A 2.5 g nanocellulose and 50 mL acetic acid were stirred for 30 min at room temperature. Next, 0.32 mL of sulfuric acid and 18 mL of acetic acid were added to the solution and stirred for 25 minutes. The solution was filtered, and then 64 mL of anhydrous acetate was added to the filtrate solution and stirred for 30 minutes. Then, the solution was precipitated for 14 h, and the precipitate was filtered by vacuum. The precipitation was then washed down to pH 7. After that, bacterial cellulose was mixed in 200 mL distilled and added 1% of TiO_2_ and 1% of graphene. The mixture was stirred for 30 minutes and then sonicated for 30 minutes. The filtrate was poured into a petri dish and dried in an oven for 24 hours at 60 C. In this study, three types of bacterial cellulose were made as follows:

1. Bacterial cellulose without adding TiO_2_ and graphene (NCB)
2. Bacterial cellulose with the addition of TiO_2_ without graphene (NCB + TiO_2_)
3. Bacterial cellulose with the addition of TiO_2_ and graphene (NCB + TiO_2_+graphene)

#### 2.1.3. Microbes Determination in Tested Water

There were two types of water samples used in this study. First, the river water flows naturally in Padang, West Sumatra. The river water was sampled at three different locations. The river water was characterized before filtration with NCB biomembrane. Second, the water was containing *E-coli* bacteria. The bacterial culturing was carried out in the laboratory. Filtering was carried out with the prepared NCB biomembrane of the two existing water samples. The effectiveness of filtration was calculated based on the ratio of microbes present in water before and after filtration [14, 15]. The experiment was repeated at least three times. The data were then processed statistically using Microsoft Excel.

## 3. Result

Figure 2 shows the results of the scanning electron microscopy (SEM) for the three types of NCB that have been conducted. Based on Figure 2, it can be shown that the addition of TIO_2_ and graphene makes the NCB surface uneven. The mixing process of TiO_2_ and graphene to the NCB induced agglomeration. In this study, a comparison has been made between NCB and NCB composites treated with TiO_2_ and graphene to remove the bacteria. TIO_2_ is the most effective catalyst for degrading organic contaminants. As a supplementary solution membrane polymer, TiO_2_ was easy to agglomerate and soluble in acetic acid. Meanwhile, adding graphene aimed to increase the ionic conductivity of the membrane. Based on the function of the additive added to NCB derived from cellulose from pineapple peel, it will be ascertained whether it can affect the effectiveness of the bacteria in the water sample.

This study aimed to clarify the NCB's effectiveness in filtering bacteria in water samples.  Table 1 shows the characteristics of the river water used in this study. Water was sampled at three different places in the city of Padang. The reason for choosing these three places was the environmental condition around the river. The first place was the river water in the refinery area close to the cement production industrial area (R1). Next, was the river basin area in Lubuk Begalung, which was close to the rubber processing industry (R2). The third was the river basin in the district Air Pacah which was close to the final waste management site in the city of Padang (R3). The observations focused on the total suspension solids (TSSs), total dissolved solids (TSSs), and pH.

Based on Table 1, it can be recognized that all samples have a similar pattern in TDS and TSS. Sample R1 had the highest TDS and TSS level, followed by the samples R3 and R2. These data follow the character of the environment around the river flow. The sample R1 was located in a cement industrial area where the distribution of cement powder was possibly very high, which may increase the TDS and TSS value in river water. Meanwhile, the samples R2 and R3 were located far from the cement industry and had lower TDS, including the TSS content. The TDS and TSS value in the sample R3 was higher than R2, possibly because of domestic waste contamination. According to the Indonesian Regulation, the samples' TDS and TSS values were high and indicated contamination. Therefore, this contamination reduction treatment needs to be carried out. Meanwhile, slightly acidic conditions were present in all samples for the pH value. The pH value also did not meet the applicable quality standards. The pH value might not be affected by the filtering process but can affect the resistance of the NCB.

The effectiveness of NCB for filtering bacteria from samples was carried out with two types of samples (river water samples and *E. Coli* bacteria culture samples).  Table 2 indicates the efficacy of river water filtration by NCB biomembranes. The filtration process was conducted by using Stainless Steel Syringe Filter Holders. The NCB biomembranes were cut and put inside the Stainless Steel Syringe Filter Holders (Figure 3). As a result, the efficacy of NCB biomembranes to filtrate the bacteria from the river water was similar. NCB biomembranes can remove more than 50% of the bacterial content in river water samples; however, TiO_2_ and graphene treatment did not significantly affect the filtering ability of bacteria from river water. Furthermore, a decrease in TDS and TSS was also detected after the filtering process, in which the filtration did not only occur in microbiological aspects but also physically and possibly chemically. Chemical testing will be carried out in another part of this study.

Table 3 presents the efficacy of *E. Coli* bacteria culture samples filtration by NCB biomembrane. Filtration of *E-coli* bacteria with NCB biomembrane has been known to eliminate more than 90% of *E-Coli* bacteria. There was an increase in the filtering ability when the filtering was only carried out for one type of bacteria. The same pattern occurred with the results of filtering with river water samples where TiO_2_ and graphene treatment had no effect on increasing the filtering effectiveness.

## 4. Discussion

The content of microbes in water samples can harm public health because they can be a source of disease [16]. Microbes contained in the water are generally in the form of bacteria, where the most common is *Escherichia coli*. These bacteria can cause diarrhea, a frightening spectre for the community [17]. Therefore, raw water that is very likely to be contaminated by microbes is highly recommended to be treated before consumption. Several techniques, including filtration (either depth filtration or surface filtration), partition and fractionation (centrifugation), and chromatography, can be used to remove microorganisms [18, 19]. Filtration is the most favoured method because it is nondestructive and nonintrusive, indicating that it will not endanger the integrity of biological materials or provoke immunological responses. Different synthetic and semisynthetic polymers have created membrane filters to attain the appropriate filtration pore size. Membrane filters are a reliable and popular technique for identifying microbial contamination in sample collection. It is one of the few conventional procedures that permit the separation of microorganisms and their subsequent determination. It also involves less planning than some other conventional approaches. Regular membrane filters cannot keep microbes because the membrane holes are too large. As a result, it is crucial to have materials better suited for microbial filtration, and research is leading to the creation of a new cellulose-based filtering medium with superior filtration characteristics.

Generally, standard commercial sterilization procedures using the microfiltration principle to remove all bacteria from heat-sensitive pharmaceutical and laboratory solutions and available water source systems can be carried out using a 0.22 *μ*m pore size filter. In general, the size of bacteria is in the range of 0.22 *μ*m to 0.45 *μ*m with the following details: *Bacillus subtilis*, *Staphylococcus aureus*, *Klebsiella pneumoniae*, and *Escherichia coli* were filtered with a pore size of 0.45 *μ*m. *Pseudomonas aeruginosa*, *Serratia marcescens*, and *Listeria monocytogenes* can be filtered with a pore size of 0.3 *μ*m and *P. aeruginosa* through a pore size filter of 0.22 *μ*m [20]. In this study, filtering with NCB made from the pineapple skin was carried out on two types of samples. The effectiveness of the type of river water sample is only 50%, which shows that there are many types of bacteria in the sample. Bacteria with large porosity will be filtered, while some will pass. These data were linear with the results of the filtering of *E. Coli*, which was able to filter more than 90% because the size of *E. Coli* is quite large.

In addition, the results showed that the NCB's porosity was most likely the only factor in the reduction of microbes in the tested water. From the perspective of microbiological content, the reinforcement of TiO_2_ and graphene was less prevalent for water purification. The previous study indicated that using TiO_2_, either with or without a combination with nanocomposites such as graphene, will provide photocatalysis for the advanced oxidation of chemical contaminants such as metals and phenols [21, 22]. Therefore, the produced NCBs should be further evaluated on water samples with heavy metals or phenol contamination characters to ensure their good effectiveness and microbes' reduction.

## 5. Conclusion

Biomembrane made from bacterial nanocellulose from the pineapple peel has been used to reduce the number of bacteria in water, especially *E. Coli*. The reinforcement of the biomembrane did not have much effect on the ability to remove existing contaminants. NCB made from the pineapple peel can be further developed for more comprehensive community water purification applications.

## Figures and Tables

**Figure 1:** The flow chart of the NCB experiment.

**Figure 2:** The SEM data of NCB and its composites.

**Figure 3:** The filtration process of samples by NCB with filtration apparatus.

**Table 1:** General characteristics of the river water.

Sample	TDS (mg/L)	TSS (mg/L)	pH
R1	2400	902	5.5
R2	500	408	5.6
R3	800	703	5.6

**Table 2:** The efficacy of river water filtration by NCB control, NCB + TiO_2_ and by NCB + TiO_2_ + graphene.

Sample	Filtration efficacy for bacteria (%)	TDS (mg/L)	TSS (mg/L)	pH
*NCB*				
R1	56.12 ± 1.60	170	350	5.5
R2	58.01 ± 1.82	190	350	5.5
R3	56.98 ± 1.88	380	360	5.6

*NCB* *+* *TIO*_*2*_				
R1	56.83 ± 1.60	170	350	5.5
R2	57.98 ± 1.52	190	350	5.5
R3	57.68 ± 1.58	380	360	5.6

*NCB* *+* *TiO*_*2*_* + graphene*				
R1	57.01 ± 1.12	170	350	5.5
R2	58.02 ± 1.91	190	350	5.5
R3	57.11 ± 1.08	380	360	5.6

**Table 3:** The efficacy of *E-coli* filtration by NCB membranes.

Sample	Filtration efficacy for *E-coli* (%)
NCB	88.85 ± 3.60
NCB-TiO_2_	90.16 ± 1.12
NCB-TIO_2_ + graphene	90.98 ± 2.51

## Data Availability

Data used to support the findings of the present study are available from the corresponding author upon request.
